The article "Statistical Analysis of COVID-19 Data for Three Different Regions in the Kingdom of Saudi Arabia: Using a New Two-Parameter Statistical Model" was published in 2022. Journal: Comput Math Methods Med.

# Statistical Analysis of COVID-19 Data for Three Different Regions in the Kingdom of Saudi Arabia: Using a New Two-Parameter Statistical Model

**DOI:** 10.1155/2022/2066787

**Published:** 2022-07-09

**Authors:** Ibrahim Al-Dayel, Mohammed N. Alshahrani, Ibrahim Elbatal, Naif Alotaibi, A. W. Shawki, Mohammed Elgarhy

**Affiliations:** ^1^Department of Mathematics and Statistics, College of Science, Imam Mohammad Ibn Saud Islamic University (IMSIU), Riyadh 11432, Saudi Arabia; ^2^Department of Mathematics, College of Science, Alkharj, Prince Sattam University, Saudi Arabia; ^3^Central Agency for Public Mobilization & Statistics (CAPMAS), Cairo, Egypt; ^4^The Higher Institute of Commercial Sciences, Al Mahalla Al Kubra, Algarbia 31951, Egypt

## Abstract

Since December 2019, the COVID-19 outbreak has touched every area of everyday life and caused immense destruction to the planet. More than 150 nations have been affected by the coronavirus outbreak. Many academics have attempted to create a statistical model that may be used to interpret the COVID-19 data. This article extends to probability theory by developing a unique two-parameter statistical distribution called the half-logistic inverse moment exponential (HLIMExp). Advanced mathematical characterizations of the suggested distribution have explicit formulations. The maximum likelihood estimation approach is used to provide estimates for unknown model parameters. A complete simulation study is carried out to evaluate the performance of these estimations. Three separate sets of COVID-19 data from Al Bahah, Al Madinah Al Munawarah, and Riyadh are utilized to test the HLIMExp model's applicability. The HLIMExp model is compared to several other well-known distributions. Using several analytical criteria, the results show that the HLIMExp distribution produces promising outcomes in terms of flexibility.

## 1. Introduction

In recent years, many various of statisticians have been attracted by create new families of distributions for example; exponentiated generalized-G in [1], logarithmic-X family of distributions [2], sine-G in [3], odd Perks-G in [4], odd Lindley-G in [5], truncated Cauchy power-G in [6], truncated Cauchy power Weibull-G-G in [7], Topp-Leone-G in [8], odd Nadarajah–Haghighi-G in [9], the Marshall–Olkin alpha power-G in [10], T-X generator studied in [11], type I half-logistic Burr X-G in [12], KM transformation family in [13], (DUS) transformation family in [14], arcsine exponentiated-X family in [15], Marshall-Olkin odd Burr III-G family in [16], among others.

Reference [17] investigates the half-logistic-G (HL-G) family, a novel family of continuous distributions with an additional shape parameter *θ* > 0. The HL-G cumulative distribution function (cdf) is supplied via

(1) $$\begin{array}{c} F\left(z;\theta ,\omega \right)=\frac{1-{\left[1-G\left(z;\omega \right)\right]}^{\theta }}{1+{\left[1-G\left(z;\omega \right)\right]}^{\theta }},\;z\in R,\theta >0. \end{array}$$

The HL-G family's density function (pdf) is described as

(2) $$\begin{array}{c} f\left(z;\theta ,\omega \right)=\frac{2\theta g\left(z;\omega \right){\left[1-G\left(z;\omega \right)\right]}^{\theta -1}}{{\left[1+{\left[1-G\left(z;\omega \right)\right]}^{\theta }\right]}^{2}},\;z\in R,\theta >0, \end{array}$$

respectively. A random variable (R.v)*Z*has pdf (2) which would be specified as*Z* ~ *HL* − *G*(*z*; *ω*).

Reference [18] presented the moment exponential (MExp) model by allocating weight to the exponential (Exp) model. They established that the MExp distribution is more adaptable than the Exp model. The cdf and pdf files are available.

(3) $$\begin{array}{c} \begin{array}{cc} G\left(t;\beta \right)=1-\left(1+\frac{t}{\beta }\right)e^{-\left(t/\beta \right)}, & t>0 \end{array}, \end{array}$$

(4) $$\begin{array}{c} \begin{array}{cc} g\left(t,\beta \right)=\frac{t}{\beta^{2}}e^{-\left(t/\beta \right)}, & t>0 \end{array}, \end{array}$$

respectively, where *β* > 0 is a scale parameter.

The inverse MExp (IMExp) distribution was presented in reference [19], and it is produced by utilizing the R.v *Z* = 1/*T*, where *T* is as follows (4). The cdf and pdf files in the IMExp distribution are specified as

(5) $$\begin{array}{c} \begin{array}{ccc} G\left(z;\beta \right)=\left(1+\frac{\beta }{z}\right)e^{-\left(\beta /z\right)}, & z>0, & \beta >0 \end{array},\\ \begin{array}{ccc} g\left(z;\beta \right)=\frac{\beta^{2}}{z^{3}}e^{-\left(\beta /z\right)}, & z>0, & \beta >0 \end{array}. \end{array}$$

In this research, we propose an extension of the IMExp model, which is built using the HL-G family and the IMExp model, known as the half-logistic inverse moment exponential (HLIMExp) distribution.

The aim goal of this article can be considered in the following items:

- To introduce a new two-parameter lifetime model which is called the HLIMExp
- The new model is very flexible, and the pdf can take different shapes such as unimodal, right skewness, and heavy tail. Also, the hrf can be increasing, upside-down, and J-shaped
- Many numerical values of the moments are calculated in Table 1. And we can note from it that (*a*) when*β* = 3and*θ*is increasing, then the numerical values of*E*(*Z*),*E*(*Z*^2^),*E*(*Z*^3^),*E*(*Z*^4^), variance(*σ*^2^), skewness (SK), and kurtosis (KU) are decreasing but the numerical values of harmonic mean (*H*) are increasing
- The simulation study is carried out to assess the behavior of parameters, and the numerical results are mentioned in Tables 2–5. From these tables, we can note that when the value of *n* is increased, the value of *Ω*1 and *Ω*4 is decreased
- Three separate sets of COVID-19 data from Al Bahah, Al Madinah Al Munawarah, and Riyadh are utilized to test the HLIMExp model's applicability. The HLIMExp model is compared to several other well-known distributions. Using several analytical criteria, the results show that the HLIMExp distribution produces promising outcomes in terms of flexibility

The following is an outline of the remainder of this article: Section 2 discusses the construction of the HLIMExp model.  Section 3 calculates the basic properties of the distribution, including the linear representation of HLIMExp pdf, order statistics, moments, moment generating function, and conditional moment. In contrast, Section 4 discusses parameter estimation using the maximum likelihood (ML) estimation method.  Section 5 employs Monte Carlo simulation techniques. In Section 6, we investigated the potentiality of the HLIMExp using three different metrics of goodness of fit such as the Akaike Information Criterion (IC) (*𝔙*1), Consistent AIC (*𝔙*2), Bayesian IC (*𝔙*3), Hannan-Quinn IC (*𝔙*4), Kolmogorov–Smirnov (*𝔙*5) test, and *p* value (*𝔙*6). Finally, Section 7 mentions the conclusion.

## 2. The New Two-Parameter Statistical Model

A nonnegative R.v *Z* with the HLIMExp model is constructed by putting (5) and (6) in (1) and (2), respectively; we should get cdf and pdf.

(6) $$\begin{array}{c} \begin{array}{cc} F\left(z;\beta ,\theta \right)=\frac{1-{\left[1-\left(1+\left(\beta /z\right)\right)e^{-\left(\beta /z\right)}\right]}^{\theta }}{1+{\left[1-\left(1+\left(\beta /z\right)\right)e^{-\left(\beta /z\right)}\right]}^{\theta }}, & z>0,\beta ,\theta >0 \end{array}. \end{array}$$

(7) $$\begin{array}{c} f\left(z;\beta ,\theta \right)=\frac{2\theta \left(\beta^{2}/z^{3}\right)e^{-\left(\beta /z\right)}{\left[1-\left(1+\left(\beta /z\right)\right)e^{-\left(\beta /z\right)}\right]}^{\theta -1}}{{\left[1+{\left[1-\left(1+\left(\beta /z\right)\right)e^{-\left(\beta /z\right)}\right]}^{\theta }\right]}^{2}},\;z>0,\theta >0. \end{array}$$

The survival function (sf) is provided by

(8) $$\begin{array}{c} \bar{F}\left(z;\beta ,\theta \right)=\frac{2{\left[1-\left(1+\left(\beta /z\right)\right)e^{-\left(\beta /z\right)}\right]}^{\theta }}{1+{\left[1-\left(1+\left(\beta /z\right)\right)e^{-\left(\beta /z\right)}\right]}^{\theta }},\;z>0,\beta ,\theta >0. \end{array}$$

The hrf or failure rate and reversed hrf for the HLIMExp are calculated as follows:

(9) $$\begin{array}{c} h\left(z;\beta ,\theta \right)=\frac{\theta \left(\beta^{2}/z^{3}\right)e^{-\left(\beta /z\right)}}{\left[1-\left(1+\left(\beta /z\right)\right)e^{-\left(\beta /z\right)}\right]\left[1+{\left[1-\left(1+\left(\beta /z\right)\right)e^{-\left(\beta /z\right)}\right]}^{\theta }\right]},\\ \tau \left(z;\beta ,\theta \right)=\frac{2\theta \left(\beta^{2}/z^{3}\right)e^{-\left(\beta /z\right)}{\left[1-\left(1+\left(\beta /z\right)\right)e^{-\left(\beta /z\right)}\right]}^{\theta -1}}{1-{\left[1-\left(1+\left(\beta /z\right)\right)e^{-\left(\beta /z\right)}\right]}^{2\theta }}. \end{array}$$

Different shapes of the pdf and hrf of HLIMExp with different parameter values are mentioned in Figures 1 and 2.

## 3. Statistical Properties

We discussed certain HLIMExp distribution features in this part, including linear representation of HLIMExp pdf, moments (Mo), the harmonic mean (**H**), moment generating function (MoGF), and conditional moment (CoMo).

### 3.1. Linear Representation

A linear form of the pdf and cdf is offered in this part to introduce statistical properties of the HLIMExp distribution. Using the following binomial expansion,

(10) $$\begin{array}{c} {\left(1+z\right)}^{-m}=\overset{\infty }{\underset{i=0}{\sum }}{\left(-1\right)}^{i}\left(\begin{array}{c} m+i-1\\ i \end{array}\right)z^{i}, \end{array}$$

where∣*z* | <1 and *b* is a positive real noninteger. By applying (10) in the next term, we get

(11) $$\begin{array}{c} {\left[1+{\left[1-\left(1+\frac{\beta }{z}\right)e^{-\left(\beta /z\right)}\right]}^{\theta }\right]}^{-2}=\overset{\infty }{\underset{i=0}{\sum }}{\left(-1\right)}^{i}\left(i+1\right){\left[1-\left(1+\frac{\beta }{z}\right)e^{-\left(\beta /z\right)}\right]}^{\theta i}. \end{array}$$

Inserting the previous equation in (7), we have

(12) $$\begin{array}{c} f\left(z;\beta ,\theta \right)=2\theta \beta^{2}\overset{\infty }{\underset{i=0}{\sum }}{\left(-1\right)}^{i}\left(i+1\right)z^{-3}e^{-\left(\beta /z\right)}{\left[1-\left(1+\frac{\beta }{z}\right)e^{-\left(\beta /z\right)}\right]}^{\theta \left(i+1\right)-1}. \end{array}$$

Again, applying the general binomial theorem, we get

(13) $$\begin{array}{c} {\left[1-\left(1+\frac{\beta }{z}\right)e^{-\left(\beta /z\right)}\right]}^{\theta \left(i+1\right)-1}=\overset{\infty }{\underset{j=0}{\sum }}{\left(-1\right)}^{j}\left(\begin{array}{c} \theta \left(i+1\right)-1\\ j \end{array}\right){\left(1+\frac{\beta }{z}\right)}^{j}e^{-\left(j\beta /z\right)}. \end{array}$$

Inserting the previous equation in (7), we have

(14) $$\begin{array}{c} f\left(z;\beta ,\theta \right)=2\theta \beta^{2}\overset{\infty }{\underset{i,j=0}{\sum }}{\left(-1\right)}^{i+j}\left(i+1\right)\left(\begin{array}{c} \theta \left(i+1\right)-1\\ j \end{array}\right)z^{-3}e^{-\left(\beta \left(j+1\right)/z\right)}{\left(1+\frac{\beta }{z}\right)}^{j}. \end{array}$$

Again, using the binomial expansion, we get

(15) $$\begin{array}{c} f\left(z;\beta ,\theta \right)=\overset{\infty }{\underset{k=0}{\sum }}S_{k}z^{-k-3}e^{-\left(\beta \left(j+1\right)/z\right)}, \end{array}$$

where

(16) $$\begin{array}{c} S_{k}=2\theta \beta^{k+2}\overset{\infty }{\underset{i,j=0}{\sum }}{\left(-1\right)}^{i+j}\left(i+1\right)\left(\begin{array}{c} j\\ k \end{array}\right)\left(\begin{array}{c} \theta \left(i+1\right)-1\\ j \end{array}\right). \end{array}$$

### 3.2. Moments

The *r*^th^ Mos of the HLIMExp distribution are discussed in this subsection. Moments are essential in any statistical study, but especially in applications, it can be used to investigate the main properties and qualities of a distribution (e.g., tendency, dispersion, skewness, and kurtosis). The *r*^th^ Mo of Z denoted by ${\overset{`}{\mu }}_{r}$ may be calculated using (8).

(17) $$\begin{array}{c} {\overset{`}{\mu }}_{r}=E\left(Z^{r}\right)=\overset{\infty }{\underset{k=0}{\sum }}S_{k}\int_{0}^{\infty }z^{r-k-3}e^{-\left(\beta \left(j+1\right)/z\right)}dz, \end{array}$$

then,

(18) $$\begin{array}{c} {\overset{`}{\mu }}_{r}=\overset{\infty }{\underset{k=0}{\sum }}S_{k}{\left(\beta \left(j+1\right)\right)}^{-r-k-2}\Gamma \left(k+r+2\right). \end{array}$$

The *r*^th^ inverse Mo of *Z* denoted by ${\overset{`}{\mu }}_{r}$ may be calculated using (8).

(19) $$\begin{array}{c} {\overset{`}{\mu }}_{r^{-1}}=E\left(Z^{-r}\right)=\overset{\infty }{\underset{k=0}{\sum }}S_{k}\int_{0}^{\infty }z^{r-k-3}e^{-\left(\beta \left(j+1\right)/z\right)}dz, \end{array}$$

then,

(20) $$\begin{array}{c} {\overset{`}{\mu }}_{r^{-1}}=\overset{\infty }{\underset{k=0}{\sum }}S_{k}{\left(\beta \left(j+1\right)\right)}^{r-k-2}\Gamma \left(k-r+2\right). \end{array}$$

The harmonic mean of *Z* is given by

(21) $$\begin{array}{c} H=E\left(\frac{1}{Z}\right)=\overset{\infty }{\underset{k=0}{\sum }}S_{k}\int_{0}^{\infty }z^{-k-4}e^{-\left(\beta \left(j+1\right)/z\right)}dz, \end{array}$$

then,

(22) $$\begin{array}{c} {\overset{`}{\mu }}_{r}=\overset{\infty }{\underset{k=0}{\sum }}S_{k}{\left(\beta \left(j+1\right)\right)}^{-k-3}\Gamma \left(r+3\right). \end{array}$$

MoGFs are useful for several reasons, one of which is their application to analysis of sums of random variables. The MoGF of *ZM*_*z*_(*t*) is deduced from (7) as

(23) $$\begin{array}{c} M_{z}\left(t\right)=\overset{\infty }{\underset{r=0}{\sum }}\frac{t^{r}}{r!}\mu_{r}^{\prime }=\overset{\infty }{\underset{r=0}{\sum }}\overset{\infty }{\underset{k=0}{\sum }}\frac{S_{k}t^{r}\Gamma \left(k-r+2\right){\left(\beta \left(j+1\right)\right)}^{r-k-2}}{r!}. \end{array}$$

Numerical values for specific values of parameters of the first four ordinary Mos, *E*(*Z*), *E*(*Z*^2^), *E*(*Z*^3^), *E*(*Z*^4^), variance (*σ*^2^), skewness (SK), and kurtosis (KU) of the HLIMExp model are reported in Table 1.

### 3.3. The Conditional Moment

For empirical intents, the shapes of various distributions, such as income quantiles and Lorenz and Bonferroni curves, can be usefully described by the first incomplete moment, which plays a major role in evaluating inequality. These curves have a variety of applications in economics, reliability, demographics, insurance, and medical. Let *Z* denote a R.v with the pdf given in (7). The *s*^th^ upper incomplete Mo say *η*_*s*_(*t*) could be expressed with

(24) $$\begin{array}{c} \eta_{s}\left(t\right)=\int_{t}^{\infty }z^{s}f\left(z;\beta ,\theta \right)dz=\overset{\infty }{\underset{k=0}{\sum }}S_{k}\int_{t}^{\infty }z^{s-k-3}e^{-\left(\beta \left(j+1\right)/z\right)}dz=\overset{\infty }{\underset{k=0}{\sum }}S_{k}{\left(\beta \left(j+1\right)\right)}^{s-k-2}\Gamma \left(k-s+2,\frac{\beta \left(j+1\right)}{t}\right). \end{array}$$

Similarly, the *s*^th^ lower incomplete Mo function is provided through

(25) $$\begin{array}{c} \phi_{s}\left(t\right)=\int_{0}^{t}z^{s}f\left(z;\beta ,\theta \right)dz=\overset{\infty }{\underset{k=0}{\sum }}S_{k}\int_{0}^{t}z^{s-k-3}e^{-\left(\beta \left(j+1\right)/z\right)}dz=\overset{\infty }{\underset{k=0}{\sum }}S_{k}{\left(\beta \left(j+1\right)\right)}^{s-k-2}\gamma \left(k-s+2,\frac{\beta \left(j+1\right)}{t}\right). \end{array}$$

## 4. Method of Maximum Likelihood

Let *z*_1_, *z*_2_, ⋯, *z*_*n*_ be a random sample of size *n* from the HLIMExp model with two parameters *β* and *θ*; the log-likelihood function is

(26) $$\begin{array}{c} L=n\ln\left(2\theta \right)-2n\ln\beta -3\overset{n}{\underset{i=1}{\sum }}z_{i}-\overset{n}{\underset{i=1}{\sum }}\frac{\beta }{z_{i}}+\left(\theta -1\right)\overset{n}{\underset{i=1}{\sum }}\log\left[G_{i}\right]-2\overset{n}{\underset{i=1}{\sum }}\log\left[1+{\left[G_{i}\right]}^{\theta }\right]. \end{array}$$

For calculation MLE estimation, we need partial derivatives of *L*(*Z* | *β*, *θ*) by parameters

(27) $$\begin{array}{c} \frac{\partial \log L}{\partial \beta }=\frac{-2n}{\beta }-\overset{n}{\underset{i=1}{\sum }}\frac{1}{z_{i}}++\left(\theta -1\right)\overset{n}{\underset{i=1}{\sum }}\frac{V_{i}}{G_{i}}-2\overset{n}{\underset{i=1}{\sum }}\frac{\theta V_{i}{\left[G_{i}\right]}^{\theta -1}}{\left[1+{\left[G_{i}\right]}^{\theta }\right]},\\ \frac{\partial \log L}{\partial \theta }=\frac{n}{\theta }+\overset{n}{\underset{i=1}{\sum }}\log\left[G_{i}\right]-2\overset{n}{\underset{i=1}{\sum }}\frac{{\left(G_{i}\right)}^{\theta }\ln\left[G_{i}\right]}{1+{\left[G_{i}\right]}^{\theta }}, \end{array}$$

where *G*_*i*_ = 1 − (1 + (*β*/*z*_*i*_))*e*^−(*β*/*z*_*i*_)^ and *V*_*i*_ = *∂G*_*i*_/*∂β* = (*β*/(*z*_*i*_)^2^)*e*^−(*β*/*z*_*i*_)^. As result, estimations of the parameters can be found ${\hat{\beta }}_{\text{MLE}}$ and ${\hat{\theta }}_{\text{MLE}}$ the solution of the two equations *∂L*/*∂β* = 0 and *∂L*/*∂θ* = 0 by using software Mathematica (9).

## 5. Simulation Results

A simulation result is included in this section to analyze the behavior of estimators in the presence of complete samples by using the Newton-Raphson iteration method and by using Mathematica (8) software. Mean square errors (*Ω*1), lower and upper bound (*Ω*2 and *Ω*3) of confidence interval (CIn), and average length (*Ω*4) of 90% and 95% are computed using Mathematica 9. The accompanying algorithm is constructed in the next part:

- 5000 RS of size *n* = 30, 50, 100, 300, 400, and 500 are generated from the HLIMExp model
- The parameters' exact values are chosen
- The ML estimates (MLEs), *Ω*1s, *Ω*2, *Ω*3, and *Ω*4 for selected values of parameters are computed
- Tables 2–5 provide the numerical outputs based on the entire data set

## 6. Applications

This section concerned with three important real data sets. The data called Saudi Arabia Coronavirus cases (COVID-19) situation in Al Bahah, Al Madinah Al Munawarah and Riyadh regions from January 2022 to May 2022.

The three data sets were obtained from the following electronic address: https://datasource.kapsarc.org/explore/dataset/saudi-arabia-coronavirus-disease-COVID-19-situation/. The data sets are reported in Table 6. The descriptive analysis of the three data sets is reported in Table 7.

Here, in this section, the three data sets mentioned below are examined to demonstrate how the HLIMExp distribution outperforms alternative models, comparing the new model to some models, namely, type II Topp-Leone inverse Rayleigh (TIITOLIR) distribution by [20], half-logistic inverse Rayleigh (HLOIR) distribution by [21], beta transmuted Lindley (BTLi) distribution by [22], the transmuted modified Weibull (TMW) distribution by [23], and the weighted Lindley (W-Li) distribution by [24]. We calculate the model parameters' MLEs and standard errors (SEs). To evaluate distribution models, we use criteria such as the *𝔙*1, *𝔙*2, *𝔙*3, *𝔙*4, *𝔙*5, and *𝔙*6 tests. In contrast, the wider distribution relates to smaller *𝔙*1, *𝔙*2, *𝔙*3, *𝔙*4, and *𝔙*5 and the highest value of *𝔙*6. The MLEs of the eight fitted models and their SEs and the numerical values of *𝔙*1, *𝔙*2, *𝔙*3, *𝔙*4, *𝔙*5, and *𝔙*6 for the three data sets are presented in Tables 8–10. We find that the HLIMExp distribution with two parameters provides a better fit than seven models. It has the smallest values of *𝔙*1, *𝔙*2, *𝔙*3, *𝔙*4, and *𝔙*5 and the greatest value of *𝔙*6 among those considered here. Moreover, the plots of empirical cdf, empirical pdf, and PP plots of our competitive model for the three data sets are displayed in Figures 3–5, respectively. The HLIMExp model clearly gives the best overall fit and so may be picked as the most appropriate model for explaining data.

## 7. Conclusion

We propose a novel two-parameter distribution called the half-logistic inverted moment exponential distribution in this research. HLIMExp's pdf may be written as a linear combination of IMExp densities. We compute explicit formulas for several of its statistical features, such as HLIMExp pdf linear representation, OS, Moms, MoGF, and CoMo. The greatest likelihood estimate is investigated. The accuracy and performance of estimations are evaluated using simulation results. Three separate sets of COVID-19 data from Al Bahah, Al Madinah Al Munawarah, and Riyadh are utilized to test the HLIMExp model's applicability. The HLIMExp model is compared to several other well-known distributions. Using several analytical criteria, the results show that the HLIMExp distribution produces promising outcomes in terms of flexibility. In the future works, we can use the new suggested model in many works such as (a) using it to study the statistical inference of the suggested model under different censored schemes, (b) using it to study the statistical inference of the suggested model under different ranked set sampling, (c) accelerated lifetime test can be studied for the new model, and (d) the statistical inference of stress strength model for the new suggested model can be studied.

## Figures and Tables

**Figure 1:** Different shapes of pdf for the HLIMExp model.

**Figure 2:** Different shapes of hrf for the HLIMExp model.

**Figure 3:** The fitted cdf, pdf, and pp plots and fitted sf of the HLIMExp model for the first data.

**Figure 4:** The fitted cdf, pdf, and pp plots and fitted sf of the HLIMExp model for the second data.

**Figure 5:** The fitted cdf, pdf, and pp plots and fitted sf of the HLIMExp model for the third data.

**Table 1:** Numerical values of Mos for the HLIMExp model for *β* = 3 different values of parameter 𝜃.

*θ*	*E*(*Z*)	*E*(*Z*^2^)	*E*(*Z*^3^)	*E*(*Z*^4^)	*H*	*σ* ^2^	SK	KU	CV
4	0.452	9.951	1.702	0.290	1.006	6.582	2.992	1.709	1.192
4.5	0.425	8.335	1.513	0.227	1.052	4.469	2.341	1.486	1.122
5	0.404	7.293	1.370	0.186	1.092	3.275	1.915	1.322	1.066
5.5	0.387	6.568	1.256	0.156	1.130	2.531	1.616	1.197	1.020
6	0.372	6.036	1.163	0.134	1.164	2.034	1.398	1.098	0.982
6.5	0.360	5.630	1.086	0.117	1.195	1.684	1.231	1.018	0.949
7	0.349	5.310	1.019	0.103	1.224	1.427	1.101	0.952	0.921
7.5	0.340	5.052	0.961	0.093	1.251	1.232	0.996	0.896	0.896
8	0.331	4.840	0.910	0.084	1.276	1.080	0.910	0.848	0.874
8.5	0.324	4.662	0.865	0.077	1.300	0.959	0.839	0.807	0.855

**Table 2:** MLEs, *Ω*1s, *Ω*2, *Ω*3, and *Ω*4 of the HLIMExp model for *β* = 0.5 and *θ* = 0.5.

*n*	MLEs	*Ω*1	90%			95%		
			*Ω*2	*Ω*3	*Ω*4	*Ω*2	*Ω*3	*Ω*4
30	0.582	0.042	0.360	0.805	0.445	0.317	0.847	0.530
	0.571	0.037	0.309	0.833	0.523	0.259	0.883	0.624
50	0.548	0.009	0.381	0.715	0.334	0.349	0.747	0.398
	0.593	0.025	0.366	0.819	0.453	0.323	0.862	0.539
100	0.550	0.005	0.419	0.680	0.261	0.394	0.705	0.311
	0.528	0.009	0.373	0.684	0.311	0.343	0.714	0.371
300	0.511	0.003	0.426	0.596	0.170	0.410	0.612	0.202
	0.496	0.005	0.391	0.601	0.211	0.371	0.621	0.251
400	0.510	0.001	0.461	0.559	0.098	0.452	0.568	0.116
	0.525	0.003	0.460	0.589	0.129	0.448	0.602	0.154
500	0.511	0.001	0.473	0.548	0.076	0.465	0.556	0.090
	0.522	0.002	0.472	0.571	0.099	0.462	0.581	0.119

**Table 3:** MLEs, *Ω*1s, *Ω*2, *Ω*3, and *Ω*4 of HLIMExp model for *β* = 0.5 and *θ* = 0.8.

*n*	MLEs	*Ω*1	90%			95%		
			*Ω*2	*Ω*3	*Ω*4	*Ω*2	*Ω*3	*Ω*4
30	0.504	0.014	0.317	0.691	0.374	0.281	0.727	0.446
	0.955	0.194	0.460	1.450	0.990	0.365	1.545	1.179
50	0.523	0.013	0.365	0.682	0.316	0.335	0.712	0.377
	0.955	0.063	0.562	1.348	0.786	0.487	1.423	0.936
100	0.524	0.006	0.401	0.647	0.245	0.378	0.670	0.292
	0.864	0.021	0.592	1.137	0.545	0.540	1.189	0.649
300	0.512	0.003	0.428	0.597	0.169	0.411	0.613	0.202
	0.840	0.011	0.652	1.028	0.376	0.615	1.064	0.448
400	0.504	0.001	0.456	0.552	0.096	0.447	0.561	0.114
	0.794	0.003	0.691	0.897	0.205	0.672	0.916	0.245
500	0.503	0.000	0.466	0.540	0.074	0.459	0.547	0.088
	0.814	0.003	0.732	0.896	0.163	0.717	0.911	0.195

**Table 4:** MLEs, *Ω*1s, *Ω*2, *Ω*3, and *Ω*4 of HLIMExp model for *β* = 0.5 and *θ* = 1.2.

*n*	MLEs	*Ω*1	90%			95%		
			*Ω*2	*Ω*3	*Ω*4	*Ω*2	*Ω*3	*Ω*4
30	0.519	0.006	0.355	0.683	0.329	0.323	0.715	0.392
	1.519	0.337	0.742	2.295	1.554	0.593	2.444	1.851
50	0.488	0.007	0.370	0.607	0.237	0.347	0.629	0.282
	1.122	0.033	0.683	1.562	0.879	0.599	1.646	1.047
100	0.507	0.005	0.420	0.595	0.175	0.403	0.612	0.209
	1.240	0.083	0.900	1.579	0.679	0.835	1.644	0.809
300	0.508	0.001	0.446	0.570	0.124	0.434	0.582	0.148
	1.244	0.032	1.002	1.485	0.484	0.955	1.532	0.576
400	0.502	0.001	0.452	0.551	0.100	0.442	0.561	0.119
	1.207	0.011	1.016	1.399	0.384	0.979	1.436	0.457
500	0.491	0.001	0.449	0.533	0.084	0.441	0.542	0.101
	1.176	0.011	1.014	1.339	0.325	0.982	1.370	0.388

**Table 5:** MLEs, *Ω*1s, *Ω*2, *Ω*3, and *Ω*4 of HLIMExp model for *β* = 1.5 and *θ* = 1.2.

*n*	MLEs	*Ω*1	90%			95%		
			*Ω*2	*Ω*3	*Ω*4	*Ω*2	*Ω*3	*Ω*4
30	1.687	0.277	1.010	2.363	1.353	0.881	2.492	1.612
	1.239	0.043	0.853	1.626	0.773	0.779	1.700	0.921
50	1.526	0.045	1.070	1.982	0.912	0.983	2.070	1.087
	1.225	0.014	0.909	1.501	0.592	0.852	1.557	0.706
100	1.529	0.032	1.206	1.852	0.646	1.144	1.914	0.770
	1.218	0.012	0.999	1.418	0.419	0.959	1.458	0.499
300	1.556	0.014	1.366	1.747	0.381	1.330	1.783	0.454
	1.215	0.006	1.121	1.369	0.249	1.097	1.393	0.297
400	1.513	0.005	1.354	1.672	0.318	1.323	1.702	0.379
	1.198	0.003	1.094	1.302	0.208	1.074	1.321	0.248
500	1.545	0.011	1.399	1.691	0.292	1.372	1.719	0.348
	1.201	0.001	1.131	1.321	0.189	1.113	1.339	0.225

**Table 6:** Al Bahah, Al Madinah Al Munawarah, and Riyadh Regions, coronavirus cases (COVID-19).

Year	Month	Coronavirus cases by regions		
		Al Bahah	Al Madinah Al Munawarah	Riyadh
2021	Jan	85	281	1994
2021	Feb	213	273	4524
2021	Mar	78	475	5612
2021	Apr	227	1001	12038
2021	May	409	2266	10458
2021	Jun	541	2167	7593
2021	Jul	772	1860	8747
2021	Aug	292	1050	3856
2021	Sep	32	193	760
2021	Oct	7	89	549
2021	Nov	6	73	401
2021	Dec	55	341	2541
2022	Jan	1430	8607	44169
2022	Feb	644	2477	19641
2022	Mar	77	460	1612
2022	Apr	49	423	691
2022	May	22	163	170

**Table 7:** Some descriptive analysis of the data.

	Al Bahah	Al Madinah Al Munawarah	Riyadh
*N*	17	17	17
Mean	290.529	1305.824	7373.882
Median	85	460	3856
Skewness	1.982	3.108	2.756
Kurtosis	4.327	10.927	8.65
Range	1424	8534	43999
Min	6	73	170
Max	1430	8607	44169
Sum	4939	22199	125356

**Table 8:** Numerical values of MLEs, SEs, *𝔙*1, *𝔙*2, *𝔙*3, *𝔙*4, *𝔙*5, and *𝔙*6 tests for the first data set.

Distributions	MLE and SE				*𝔙*1	*𝔙*2	*𝔙*3	*𝔙*4	*𝔙*5	*𝔙*6
	*α*	*β*	*θ*	*λ*						
HLIMExp		24.214	0.336		231.459	232.317	229.92	231.625	0.167	0.732
		(9.688)	(0.081)							
TIITOLIR	6.626	0.196			236.208	237.065	234.669	236.373	0.244	0.265
	(1.828)	(0.051)								
HLOIR	8.739	0.272			233.253	234.11	231.714	233.419	0.204	0.48
	(2.643)	(0.059)								
W-Li	0.088	0.004			232.468	233.326	230.929	232.634	0.275	0.153
	(0.078)	(0.001)								
BT-Li	0.010	0.320	0.359	0.383	232.376	235.709	229.297	232.707	0.181	0.631
	(0.017)	(0.568)	(0.138)	(1.139)						
TMW	0.230	0.00000001	0.0027	0.481	235.812	241.267	231.965	236.226	0.243	0.27
	(0.140)	(0.00002)	(0.0011)	(0.496)						
ILBE	70.429				263.621	263.888	262.851	263.704	0.427	0.004109
	(12.078)									
LBE	145.265				247.564	247.831	246.794	247.647	0.321	0.06
	(24.913)									

**Table 9:** Numerical values of MLEs, SEs, *𝔙*1, *𝔙*2, *𝔙*3, *𝔙*4, *𝔙*5, and *𝔙*6 tests for the second data set.

Distributions	MLE and SE				*𝔙*1	*𝔙*2	*𝔙*3	*𝔙*4	*𝔙*5	*𝔙*6
	*α*	*β*	*θ*	*λ*						
HLIMExp		292.561	0.520		276.46	277.317	274.921	276.626	0.118	0.972
		(103.158)	(0.138)							
TIITOLIR	89.906	0.311			278.671	279.528	277.132	278.837	0.163	0.755
	(20.808)	(0.085)								
HLOIR	114.890	0.412			277.112	277.969	275.573	277.278	0.125	0.954
	(29.837)	(0.095)								
W-Li	0.053	0.0008			282.778	283.635	281.239	282.943	0.288	0.119
	(0.075)	(0.0002)								
BT-Li	0.001	0.496	0.478	0.663	284.572	287.905	281.494	284.903	0.358	0.026
	(0.002)	(0.726)	(0.225)	(1.037)						
TMW	0.519	0.00000004	0.0006	0.669	286.033	291.488	282.185	286.447	0.239	0.286
	(0.400)	(0.00002)	(0.0002)	(0.376)						
ILBE	596.909				284.757	285.023	283.987	284.84	0.291	0.112
	(102.369)									
LBE	652.912				294.272	294.539	293.503	294.355	0.272	0.16
	(111.973)									

**Table 10:** Numerical values of MLEs, SEs, *𝔙*1, *𝔙*2, *𝔙*3, *𝔙*4, *𝔙*5, and *𝔙*6 tests for the third data set.

Distributions	MLE and SE				*𝔙*1	*𝔙*2	*𝔙*3	*𝔙*4	*𝔙*5	*𝔙*6
	*α*	*β*	*θ*	*λ*						
HLIMExp		822.893	0.377		339.578	340.435	338.039	339.744	0.158	0.788
		(320.841)	(0.093)							
TIITOLIR	224.204	0.218			344.149	345.006	342.61	344.314	0.216	0.407
	(59.549)	(0.058)								
HLOIR	292.158	0.299			341.443	342.3	339.904	341.609	0.178	0.653
	(84.846)	(0.065)								
W-Li	0.020	0.0001			341.224	342.082	339.685	341.39	0.2	0.506
	(0.041)	(0.00003)								
BT-Li	0.00032	0.859	1.157	0.229	365.36	368.694	362.282	365.692	0.319	0.064
	(0.00007)	(0.103)	(0.337)	(0.385)						
TMW	0.302	0.00000027	0.0001	0.619	345.244	350.698	341.396	345.658	0.179	0.648
	(0.177)	(0.00008)	(0.00004)	(0.425)						
ILBE	2175				363.338	363.605	362.569	363.421	0.419	0.0051
	(372.994)									
LBE	3687				356.487	356.753	355.717	356.569	0.281	0.1360
	(632.305)									

## Data Availability

All data are mentioned in this article.
